# MicroRNA-34/449 targets IGFBP-3 and attenuates airway remodeling by suppressing Nur77-mediated autophagy

**DOI:** 10.1038/cddis.2017.357

**Published:** 2017-08-10

**Authors:** Huiming Yin, Shu Zhang, Yahong Sun, Sha Li, Yunye Ning, Yuchao Dong, Yan Shang, Chong Bai

**Affiliations:** 1 Department of Respiration, First Affiliated Hospital, Hunan University of Medicine, Huaihua 418000, China; 2 Department of Respiratory Medicine, Seventh People's Hospital of Shanghai University of TCM, Shanghai 200137, China; 3 Department of Respiratory Medicine, Zhejiang Haining People's Hospital, Zhejiang Haining 314400, China; 4 Department of Respiratory and Critical Care Medicine, Changhai Hospital, Second Military Medical University, Shanghai 200433, China

## Abstract

Autophagy plays critical roles in airway inflammation and fibrosis-mediated airway remodeling and many factors including proinflammatory cytokines and inflammation related pathways are involved in the process. The aim of the present study was to examine the role of epithelial microRNAs (miRNAs) in autophagy-mediated airway remodeling and to identify the factors involved and the underlying mechanisms. Serum miR-34/449, inflammatory factors, and autophagy and fibrosis-related proteins were determined by real-time PCR, enzyme-linked immunosorbent assay and western blotting in 46 subjects with asthma and 10 controls and in the lung epithelial cell line BEAS-2B induced with IL-13 and treated with miRNA mimics. Luciferase assays were used to verify IGFBP-3 as a target of miR-34/449, and immunohistochemistry, immunofluorescence and co-immunoprecipitation were used *in vitro* and *in vivo* study. miR-34/449 were downregulated in patients with asthma in parallel with the upregulation of autophagy-related proteins. Proinflammatory factors and fibrosis-related proteins were significantly higher in asthma patients than in healthy controls. IL-13 induction promoted autophagy and upregulated miR-34/449 in BEAS-2B cells, and these effects were restored by IGFBP-3 silencing. miR-34/449 overexpression suppressed autophagy, decreased fibrosis, activated Akt, downregulated fibrosis-related factors, and downregulated proinflammatory cytokines and nuclear factor *κ*B by targeting IGFBP-3. *In vivo* experiments showed that miR-34/449 overexpression was associated with Nur77 nuclear translocation and IGFBP-3 downregulation in parallel with decreased airway remodeling by decreased autophagy. miR-34/449 are potential biomarkers and therapeutic targets in asthma. miR-34/449 may contribute to airway inflammation and fibrosis by modulating IGFBP-3 mediated autophagy activation.

Asthma is an inflammatory disease of the airways characterized by infiltration of inflammatory factors such as eosinophils, lymphocytes, and mast cells and reversible broncho-constriction.^1^ Over time, the secreted factors and cytokines induce mucous cell metaplasia, angiogenesis and subepithelial fibrosis, leading to structural remodeling of the airways.^2^ Authophagy, a highly conserved catabolic mechanism for the lysosomal degradation of proteins and organelles, has been linked to inflammatory diseases, and autophagy is associated with asthma through genetic and immune mechanisms and because of the role of autophagy in fibrosis and airway remodeling.^3, 4^ Autophagy involves the p62/sequestosome, an autophagic receptor that functions as a signaling molecule for various pathways including nuclear factor *κ*B (NF-*κ*B) and mTOR.^5^ P62 is an autophagic adapter that interacts with the autophagosomal marker LC3, which exists in two forms, LC3-I and LC3-II. Conjugation of LC3-I to phosphatidylethanolamine results in the formation of LC3-II, which is recruited to autophagosomal membranes and degraded by the lysosome.^6^ The ratio of LC3-II to LC3-I reflects the formation of autophagosomes and is therefore a marker of autophagy. Autophagy is modulated by cytokines, and the cytokine interleukin (IL)-13, which is associated with autophagy, plays an important role in asthma by regulating IgE synthesis, mucus hypersecretion, airway hyper-responsiveness and fibrosis.^7^

Insulin growth factor binding protein-3 (IGFBP-3), which modulates the activity of IGF and is involved in many human diseases, plays a role in the pathogenesis of asthma by modulating the tumor necrosis factor (TNF)-*α* induced expression of NF-*κ*B signaling pathway molecules, suggesting that IGFBP-3 plays a role in airway inflammation and hyper-responsiveness through an IGF-independent pathway.^8^ The NF-*κ*B signaling pathway is activated in asthma, and Nur77 (also known as NR4A1), a transcription factor that regulates many biological processes including inflammation and immunity, inhibits the NF-*κ*B pathway in lung epithelial cells.^9^ Translocation of Nur77 from the nucleus to the cytosol or mitochondria results in apoptosis or autophagy.^10^ Nur77 deficiency resulted in increased mucus cell hyperplasia and airway inflammation in a murine model of ovalbumin (OVA)-induced airway inflammation, suggesting that Nur77 plays a protective role against airway inflammation.

MicroRNAs (miRNAs) are small non-coding RNAs that regulate the expression of target genes by binding to the 3′ untranslated region (3′-UTR) of their promoters, suppressing translation or inducing degradation.^11^ miRNAs are involved in many biological and pathological processes including inflammation through the modulation of their target genes, and they play a role in the pathogenesis of allergic inflammatory diseases including asthma.^12^

In the present study, we examined the role of miR-34/449 and autophagy in airway inflammation and remodeling in a cohort of patients with asthma, in IL-13 induced lung epithelial cells *in vitro*, and in a murine model of OVA-induced airway inflammation *in vivo* and explored the underlying mechanisms.

## Results

### Serum levels of miR-34 and miR-449 and autophagy-related proteins in asthma patients or OVA-induced asthma mouse

Table 1 shows the clinicopathological characteristics of the 46 patients with asthma and 10 healthy controls included in the analysis. Bioinformatics analysis using Targetscan showed that IGFBP-3 is a potential target of miR-34 and miR-449. We therefore focused our analysis on these two miRNAs. Real-time PCR analysis of miR-34 and miR-449 showed that the levels of the two miRNAs were significantly lower in asthma patients than in healthy controls (Figures 1a and b). Western blot analysis of autophagy-related proteins and densitometric quantification showed that the LC3-II/LC3-I ratio and Beclin-1 expression were significantly higher, whereas P62 protein expression was significantly lower in the serum of asthma patients than in that of healthy controls (Figures 1c–f). The levels of inflammatory factors (IL-5, IL-6, IL-13, and TNF-*α*) and those of fibrosis-related proteins (basic fibroblast growth factor (bFGF), IGFBP-3, and TGF-*β*) were significantly higher in asthma patients than in healthy controls (Table 1).

We also found that the expression of miR-34 and miR-449 were decreased in both serum and lung tissues from OVA-induced asthma mouse (Figures 1g–j). So, it is reliable to use OVA-induced asthma mouse model in this study.

### IGFBP-3 knockdown inhibited IL-13 induced autophagy and miR-34/449 upregulation

To examine the association between IGFBP-3 and autophagy in airway inflammatory responses, BEAS-2B human bronchial epithelial cells were transfected with siRNA against IGFBP-3, which resulted in a significant inhibition of IGFBP-3 mRNA and protein expression (Figure 2a). Silencing of IGFBP-3 reversed the IL-13 induced increase in the LC3-II/LC3-I ratio and Beclin-1 upregulation, as well as P62 downregulation (Figures 2b–e),indicating that autophagy induced by IL-13 in lung epithelial cells is mediated by IGFBP-3. IGFBP-3 knockdown also abolished the IL-13 induced downregulation of miR-34 and miR-449 in epithelial cells (Figures 2f and g). IGFBP-3 knockdown had no effect on IL-13 induced upregulation of Bcl-2 and Nur77 (Figure 2h–j). However, co-immunoprecipitation experiments showed that Nur77 interacts with Bcl-2, abolishing the IL-13 induced upregulation of Beclin-1 (Figure 2k).

### Effect of miR-34/449 overexpression on IL-13 induced epithelial cell inflammation mediated by IGFBP-3 and Nur77 subcellular localization

To examine the role of miR-34 and miR-449 in IL-13 induced airway inflammation mediated by IGFBP-3, the two miRNAs were overexpressed by transfection of miR mimics into BEAS-2B cells (Figures 3a and b). Overexpression of miR-34 and miR-449 significantly downregulated IGFBP-3 in the presence or absence of IL-13 induction (Figures 3c and d), significantly activated Akt, as determined by the ratio of phospho-Akt to Akt (Figures 3e–g), and promoted Nur77 nuclear translocation in response to IL-13 induction (Figures 3h–j). Immunofluorescence analysis confirmed that miR-34 and miR-449 promoted Nur77 nuclear translocation in response to IL-13 induction (Figure 3k). Taken together, these results indicated that miR-34 and miR-449 promote Nur77 nuclear translocation by downregulating IGFBP-3 in association with epithelial cell inflammation.

### miR-34/449 overexpression inhibited IL-13 induced autophagy and decreased BEAS-2B cell fibrosis and inflammation

The effects of miR-34/449 on IL-13-induced autophagy were examined next. The results showed that overexpression of miR-34/449 suppressed IL-13-induced autophagy, similar to the effect of the autophagy inhibitor 3-MA (Figures 4a–d). Furthermore, the IL-13 induced upregulation of the fibrosis markers bFGF, collagen I and II, and *α*-smooth muscle actin (*α*-SMA) was inhibited by miR-34/449 overexpression to a level similar to that induced by 3-MA (Figures 4e–i), indicating that miR-34/449 downregulation is involved in autophagy-mediated fibrosis associated with airway inflammation. Similarly, miR-34/449 overexpression suppressed the IL-13-induced upregulation of the IL-5, IL-6 and TNF-*α* cytokines (Figures 5a–d), and the proinflammatory transcription factor NF-*κ*B (Figures 5e and f) to a level similar to that induced by the autophagy inhibitor 3-MA, suggesting that miR-34/449 are involved in autophagy-induced inflammation in epithelial cells.

### IGFBP-3 is a target of miR-34/449

Figure 6a shows the alignment and complementarity between miR-34/449 and the seed sequence in the 3′-UTR of human IGFBP-3. A dual luciferase assay showed that co-transfection with miR-34/449 mimics decreased the luciferase activity of the wild-type, but not that of the mutant 3′-UTR of IGFBP-3, confirming that IGFBP-3 is a target of miR-34 and miR-449 (Figures 6b and c).

### miR-34/449 overexpression decreased OVA-induced airway remodeling by suppressing autophagy-mediated airway inflammation and fibrosis *in vivo*

*In vivo* experiments in a murine model of OVA-induced airway inflammation showed that miR-34/449 overexpression suppressed the OVA-induced upregulation of IL-5, IL-6 and TNF-*α* in bronchoalveolar lavage fluid (BALF) similar to autophagy inhibition, as determined by enzyme-linked immunosorbent assay (ELISA; Figures 7a–c). Masson’s trichrome staining and immunohistochemical analysis of lung tissues showed that miR-34/449 overexpression inhibited OVA-induced pulmonary fibrotic changes and *α*-SMA expression, respectively, similar to treatment with 3-MA (Figures 7d and e). Similar results were obtained by immunofluorescence analysis of TGF-*β* and western blot analysis of bFGF, collagen I, collagen III and *α*-SMA (Figures 7f–k). Taken together, these results indicated that miR-34/449 mediate autophagy-induced airway inflammation and fibrosis *in vivo*.

### Effect of miR-34/449 and its target IGFBP-3 on Nur77 distribution and autophagy *in vivo*

The effect of miR-34/449 on the activity of Nur77 was examined in our mouse model of OVA-induced airway inflammation. Immunofluorescence analysis showed that miR-34/449 overexpression promoted Nur77 nuclear translocation in parallel with the downregulation of IGFBP-3 as shown by western blotting in total cell lysates, similar to the effect of 3-MA. The results also showed that inhibition of IGFBP-3 mediated autophagy activation suppressed NF-*κ*B expression, which can impact the expression of inflammation-related factors. (Figures 8a–e). miR-34/449 overexpression also decreased the LC3-II/LC3-I ratio and downregulated Beclin-1, although it had no significant effect on P62 expression *in vivo* (Figures 8f–i). Taken together, these results indicated that miR-34/449 modulate autophagy and mediate airway inflammation and fibrosis, promoting the nuclear translocation of Nur77 by downregulating IGFBP-3 and resulting in the inhibition of NF-*κ*B mediated inflammation.

## Discussion

Asthma is an inflammatory disorder that involves several molecular and cellular processes, among which autophagy plays an important role in mediating allergic inflammation.^3^ miRNAs are involved in inflammatory responses through the genes that they regulate, and several differentially expressed miRNAs have been identified in asthma.^13^ In the present study, we examined the role of miR-34 and miR-449 and their target IGFBP-3 in airway inflammation and remodeling associated with autophagy using an IL-13 induced airway inflammation model *in vitro* and an OVA-induced mouse model of allergic asthma *in vivo*.

Analysis of 46 asthmatic patients and 10 controls showed that miR-34 and miR-449 were downregulated in the serum of patients with asthma concomitant with the upregulation of autophagy-related proteins and increased levels of proinflammatory factors and fibrosis-related proteins. Members of the miR-34/449 family were previously identified among differentially expressed miRNAs in patients with asthma, as determined by microarray analysis, and miR34/449 were downregulated in response to IL-13 stimulation in cultured bronchial epithelial cells.^14^ miR-449 regulates the differentiation of ciliated epithelial cells by downregulating its target NOTCH1.^15^ Several other miRNAs have been identified for their involvement in allergic airway inflammation, including miR-let-7, miR-155 and miR-126.^16, 17, 18^ The miRNA let-7 inhibits IL-13 expression, and silencing of let-7 inhibits cytokine production and attenuates disease symptoms in an animal asthma model. miRNAs have been studied as targets for the treatment of allergic diseases, and suppression of miR-126 reduces inflammation, airway hyper-responsiveness, eosinophil recruitment and mucus hypersecretion, inhibiting the asthma phenotype.^19^

The involvement of autophagy in the pathogenesis of asthma was demonstrated previously by microscopic examination showing autophagosome formation in fibroblasts from asthmatic patients.^20^ Furthermore, airway remodeling and loss of lung function in asthma have been linked to genetic variants in the autophagy-related gene Atg5.^21^ A recent study showed that increased airway responsiveness and inflammatory cytokine expression in BALF were associated with LC3 upregulation and increased autophagosome formation in eosinophils in an OVA-induced asthma mouse model, suggesting the involvement of autophagy in allergic inflammation.^3^ The results of the present study showed that autophagy was increased in asthma patients compared with that in healthy controls and induced by IL-13 treatment in lung epithelial cells. Furthermore, miR-34/449 overexpression suppressed IL-13 induced autophagy and decreased lung fibrosis similar to the effect of the autophagy inhibitor 3-MA, confirming that the effects of miR-34/449 on airway inflammation and pulmonary remodeling associated with asthma are mediated at least in part by the activation of autophagy.

The roles of miR-34/449 and autophagy in airway inflammation were investigated in human lung epithelial BEAS-2B cells treated with IL-13, which showed that autophagy was mediated by the IGF-I binding protein IGFBP-3. IGFBP-3 was previously shown to be downregulated in the lungs of OVA-induced asthmatic mice and to inhibit airway inflammation through crosstalk with the NF-*κ*B signaling pathway.^22^ Recombinant IGFBP-3 was shown to have a protective effect against allergic airway inflammation through the modulation of vascular endothelial growth factor expression.^8^ The effects of IGFBP-3 are mediated by IGF dependent and independent pathways, and its antiproliferative action has been studied in cancer cells and shown to be associated with the modulation of angiogenesis.^23^ IGF-I promotes fibrosis, airway inflammation and hyper-responsiveness through interaction with inflammatory mediators, and IGFBP-3 blocks these effects possibly by sequestering IGF-I and inhibiting its activity.^24^ Because IGFBP-3 decreases airway inflammation and airway hyper-responsiveness it has been studied extensively as a potential therapeutic target for the treatment of asthma. We identified IGFBP-3 as a direct target of miR-34/449 and showed that inflammatory responses and airway fibrosis associated with asthma may be mediated by the modulation of IGFBP-3 and its effects on the regulation of autophagy.

In the present study, the IL-13-mediated induction of autophagy occurred in parallel with the upregulation of Nur77, and IGFBP-3 downregulation by miR-34/449 activated Akt, suppressed the IL-13 induced upregulation of proinflammatory factors and NF-*κ*B, and promoted Nur77 nuclear translocation in response to IL-13 induction. IGFBP-3 associates with Nur77 in the cytoplasm, and Nur77 induces cell death possibly by interacting with Bcl-2, promoting the release of Beclin-1 and the induction of autophagy.^25, 26^ Our co-immunoprecipitation experiments showed that Nur77 interacted with Bcl-2, suggesting that a similar mechanism may be involved in the induction of autophagy and airway remodeling in asthma. Nur77 was suggested to play a protective role in airway inflammation mediated by the inhibition of NF-*κ*B activity.^9^ The present results support the protective role of Nur77, as the nuclear localization of Nur77 occurred in parallel with decreased inflammation and NF-*κ*B expression. These results were confirmed *in vivo*, as Nur77 nuclear translocation was associated with the downregulation of IGFBP-3 and NF-*κ*B, and the downregulation of fibrosis factors and decreased airway remodeling in our OVA-induced model of asthma.

In conclusion, we showed that airway inflammation involves the induction of autophagy, which may be associated with the downregulation of miR-34/449, leading to the upregulation of their target IGFBP-3, the translocation of Nur77 from the nucleus to mitochondria, decreased Akt signaling, and increased fibrosis. These findings shed light on the mechanisms underlying airway inflammation and identify novel potential targets for the treatment of asthma and other inflammatory diseases of the airways.

## Materials and methods

### Ethics statement

All experimental procedures were carried out in strict accordance with the international and national guidelines and were approved by the Changhai Hospital Affiliated to the Second Military Medical University Ethics Committee. All protocols were performed under conditions to minimize animal suffering.

### Reagents

Chicken egg OVA was purchased from Sigma (St. Louis, MO, USA); 3-Methyladenine (3-MA) and TRIzol were purchased from Gibco-BRL (Grand Island, NY, USA). The PCR kit was obtained from Promega (Madison, WI, USA). All antibodies were purchased from Santa Cruz Biotechnology, Inc. (Santa Cruz, CA, USA). Other laboratory reagents were obtained from Sigma.

### Clinical specimen collection

Serum samples from 46 asthma patients or 10 healthy volunteers were obtained at the Changhai Hospital Affiliated to the Second Military Medical University between July 2015 and October 2016. The patients included 18 men and 28 women. Thirteen patients were diagnosed with well differentiation, 12 and 21 patients were moderate, and poor differentiation as categorized clinically,^27^ respectively. The diagnosis of lung adenocarcinoma was confirmed by qualified clinical pathologists. All the specimens were frozen in liquid nitrogen immediately after resection. This study was approved by the Changhai Hospital Affiliated to the Second Military Medical University and written informed consent was obtained from all patients.

### BEAS-2B cell culture and viability

The human lung epithelial BEAS-2B cell line (purchased from Procell Life Science Co., Ltd., China) was cultured at 37 °C in a humidified atmosphere with 5% CO_2_ in Dulbecco’s modified Eagle’s medium/F12 medium supplemented with 10% fetal bovine serum, 100 U/ml penicillin and 100 ng/ml streptomycin (Invitrogen, Tokyo, Japan). To induce airway fibrosis and inflammation, BEAS-2B cells transfected with/without MiR-34/449 mimics or siRNA against IGFBP-3 were stimulated with 20 ng/ml IL-13 for up to 72 h. Non-IL-13-treated cells were incubated under the same conditions as the controls.

### Plasmid constructs

To knockdown IGFBP-3 expression, siRNA against IGFBP-3 (siIGFBP-3) was constructed as follows: siIGFBP-3 (5′-CTGCTGGTGTGTGGATAAGTATG-3′). The sequences (including the scramble negative siRNA) were chemically synthesized (Genechem, Shanghai, China) and subcloned into the pENTR vector (Invitrogen, Carlsbad, CA, USA).

### Luciferase reporter assay

To construct luciferase reporter vectors, cDNA fragments of the 3′-UTR of IGFBP-3 containing the predicted potential miR-43 and miR-449 binding sites were amplified by PCR and subcloned downstream of the luciferase gene in the pGL3 luciferase vector (Ambion, Inc., Austin, TX, USA) after *Bgl* II/*Xho* I restriction enzyme digestion. The 3′-UTR of IGFBP-3 (containing the binding sites for miR-43 or miR-449) was amplified from a cDNA library with the following primers: forward, 5′-GGCTAGCCAGGAAGCGGGGCTTC-3′ and reverse, 5′-GCTCGAGCTTGGCAGTCTTTTGTGCAAAATA-3′.

The mutant IGFBP-3 3′-UTR (four nucleotides were mutated in the binding sites) primer sequences were as follows: forward, 5′-GGCTAGCCAGGAAGCGGGGCTTC-3′ and reverse, 5′-GCTCGAGCTTGG**GTCA**CTTTTGTGCAAAATA-3′.

For luciferase assays, cells were cultured in 24-well plates and co-transfected with 50 ng of the corresponding vectors containing firefly luciferase together with 25 ng of miR-34/449 mimics or control (GenePharma, Shanghai, China). Transfection was performed using Lipofectamine 2000 (Invitrogen). At 48 h post-transfection, relative luciferase activity was calculated by normalizing the Firefly luminescence to the Renilla luminescence using a Dual-Luciferase Reporter Assay (Promega) according to the manufacturer’s instructions.

### Murine model of OVA-induced asthma

Male BALB/c mice (6–8 weeks old, weighing 18–24 g) for the asthma model were obtained from the Shanghai SLAC Laboratory Animal Co., Ltd. The asthmatic model was established by treatment with OVA. The mice were sensitized on days 0, 7 and 14 by intraperitoneal injection of 20 *μ*g OVA emulsified in 1 mg aluminum hydroxide in a total volume of 0.2 ml. Seven days after the last sensitization, the mice were exposed to 1% OVA aerosol for up to 1 h every day for 7 days. The 1% OVA aerosol was generated by a compressed air atomizer driven by filling a Perspex cylinder chamber (diameter 50 cm, height 50 cm) with a nebulized solution. Saline was used in the control group instead of OVA. Mice were killed under anesthesia with sodium pentobarbital (50 mg/kg). The trachea was cannulated, and both lungs and airways were rinsed in 1 ml PBS for the collection of BALF. The right lungs were collected, frozen in liquid nitrogen and kept at −80 °C until used for western blotting. The left lungs were preserved and fixed in 4% paraformaldehyde, and then used for immunohistochemical analyses. All animal studies were performed in accordance with the Guide for the Care and Use of Laboratory Animals. All study protocols were approved by the Ethics Committee of Changhai Hospital Affiliated to the Second Military Medical University.

### Treatment protocol

All drugs were administered before the secondary challenge: 15 mg/kg 3-methyladenine (3-MA) was injected intraperitoneally in mice 30 min before the secondary OVA challenges on days 7–28. Control mice were intraperitoneally injected with PBS. In addition, a total of 10 doses of miR-449 and miR-34 were administered every 3 days (dissolved in RNA-free water and then given intranasally in a volume of 15 *μ*l) before the secondary OVA challenges on days 7–28.

### Masson trichrome staining

For the histological analyses, lung specimens obtained at the end of the experiments were fixed in 10% buffered paraformaldehyde. The paraffin-embedded lung specimens were cut into 5*-μ*m-thick sections, deparaffinized, and stained with Masson trichrome for the light microscopic visualization of collagen fibers and muscle fibers. The stained tissue sections were examined using an optical microscope system, and five images were taken for each section.

### Immunofluorescence microscopy

BEAS-2B cells or lung tissues were washed in PBS and fixed in 4% paraformaldehyde. After blocking with 3% BSA, cells or tissue slices were incubated with the primary antibodies mouse anti-TGF-*β* and mouse anti-Nur77 for 1 h at 37 °C, followed by incubation with secondary antibodies (FITC-conjugated anti-mouse IgG) for 1 h. DAPI (1 *μ*g/ml) was used for nuclear tracking. Morphological changes were observed by fluorescence microscopy, and the intracellular distribution of Nur77 and the location of the nucleus were determined using a confocal laser scanning microscope (TCSNT; Leica, Deerfield, IL, USA).

### Western blot analysis

Western blot analysis was performed using cell lysates or tissue homogenates in urea buffer (8 M urea, 1 M thiourea, 0.5% CHAPS, 50 mM dithiothreitol and 24 mM spermine). Cytoplasmic and nuclear protein fractions were prepared using NE-PER nuclear and cytoplasmic extraction reagents (Pierce, USA), respectively, following manufacturer’s protocols. *β*-tubulin was used as a loading control for the cytoplasmic fraction, whereas PARP was used as a loading control for the nuclear fraction. Samples (40 *μ*g total protein) were separated by SDS-PAGE and transferred to nitrocellulose membranes (Millipore, MA, USA). After blocking in 5% nonfat milk for 1 h, the membranes were incubated with primary antibodies against Nur77 (1:1000), IGFBP-3 (1:200), Akt (1:200), p-Akt (1:200), Bcl-2 (1:400), Beclin-1 (1:300), LC3 (1:400), P62 (1:200), *β*-tubulin (1:800), PARP (1:500), IL-5 (1:400), IL-6 (1:400), TNF*α* (1:200), NF-*κ*B (1:200), *β*-tubulin (1:1000), *α*-SMA (1:1000) and GAPDH (1:2000) at 4 °C overnight. All primary antibodies were from Santa Cruz Biotechnology. After washing, the membranes were incubated with horseradish peroxidase-conjugated secondary antibodies for 1 h at room temperature. Signals were detected using an ECL detection system (GE Healthcare, USA) and analyzed by ImageJ 1.42q software (National Institutes of Health).

### Immunoprecipitation

Cells were lysed in 20 mM Tris-HCl (pH 7.5) containing 1 mM EDTA, 1 M KCl, 5 mM MgCl_2_, 10% glycerol (v/v), 1% Triton X-100 (v/v), 0.05% 2-mercaptoethanol (v/v) and protease, and phosphatase inhibitors. The cell lysates (1–4 mg) were pre-cleared with protein G beads at 4 °C for 30 min and subsequently incubated with protein G beads pre-bound with antibody at 4 °C for 2–16 h. The beads were washed three times with 1% NP40, mixed with 6 × sample buffer, and subjected to SDS-PAGE and immunoblotting.

### Quantitative RT-PCR

To determine the mRNA levels of the target genes, total RNA was extracted from the clinical serum, cells or tissues using the Trizol reagent (Invitrogen). Reverse transcription reactions were performed using 5 *μ*g of total RNA following the standard protocol supplied with the SYBR Premix Ex Taq II (TaKaRa, Daliang, China). The resulting cDNA was used for PCR, and GAPDH was used as a loading control. All the reactions had a hot start of 5 min at 9 °C and a final elongation step at 72 °C for 10 min. The primers used were as follows: GAPDH, 5′-ATGGGGAAGGTGAAGGTCG-3′ (sense) and 5′-GGGGTCATTGATGGCAACAATA-3′ (antisense); miR-34, 5′-GGCAGTGTCTTAGCTGGTTGT-3′ (sense) and 5′-TGGTGTCGTGGAGTCG-3′ (antisense); miR-449, 5′-ACACTCCAGCTG GGTGGCAGTGTATTGTTA-3′ (forward) and 5′-TGGTGTCGTGGAGTCG-3′ (reverse); U6, 5′-CTCGCTTCGGCACA-3′ (sense) and 5′-AACGCTTCACGAATTTGCGT-3′ (antisense). Amplified products were separated on agarose gels, visualized and quantified using a thermostated Cary 300 UV-Vis spectrophotometer (Varian, Sunnyvale, CA, USA).

### Detection of soluble inflammatory cytokines by ELISA

To examine the amount of IL-6, IL-13, IL-1*β* and TNF-α in the serum, BALF or the supernatant of BEAS-2B cells, commercially available ELISA kits (Sen-Xiong Technology, Shanghai, China) were used. In accordance with the manufacturer’s instructions, all serum or supernatants were stored at −80 °C before measurements were taken, and both the standards and samples were run in triplicate. The OD_450_ was calculated by subtracting the background value, and standard curves were plotted.

### Statistical analysis

All data were expressed as the mean±S.D. Data analysis was performed using the GraphPad Prism 6.0 software. When analyzing two groups, Student’s *t*-tests were used to identify statistical significance. When comparing multiple groups, one-way analysis of variance followed by Tukey’s multiple comparisons tests were used to determine statistical differences. A value of *P*<0.05 was considered significant.

## Figures and Tables

**Figure 1:** Expression levels of miR-34/449 and autophagy-related proteins in asthma patients or OVA mouse. (**a** and **b**) Real-time PCR measurement of miR-34 (**a**) and miR-449 (**b**) expression in the serum from asthma patients and healthy controls. Values represent the mean±S.E.M. (*n*=5), *P<0.05, **P<0.01, ***P<0.001 *versus* normal control. (**c**–**f**) Western blot analysis of Beclin-1, LC3 and P62 in airway tissues from normal and patient groups and densitometric quantification of bands. Values represent the mean±S.E.M. (*n*=5), ***P<0.001 *versus* normal control. (**g** and **h**) Real-time PCR measurement of miR-34 (**g**) and miR-449 (**h**) expression in the serum from OVA-induced asthma mouse and healthy controls. Values represent the mean±S.E.M. (*n*=5), ***P<0.001 *versus* normal control. (**i** and **j**) Real-time PCR measurement of miR-34 (**i**) and miR-449 (**j**) expression in the tissue from OVA-induced asthma mouse and healthy controls lung tissue. Values represent the mean±S.E.M. (*n*=5), ***P<0.001 *versus* normal control

**Figure 2:** IL-13-induced autophagy is dependent on IGFBP-3 expression. BEAS-2B cells were transfected with siRNA against IGFBP-3 or scrambled siRNA (SCR) for 72 h. (**a**) The expression of IGFBP-3 was assessed by western blotting and real-time PCR. Values represent the mean±S.E.M. (*n*=5), ***P<0.001 *versus* control. (**b**–**k**) BEAS-2B cells transfected with siIGFBP-3 or SCR were treated with or without 20 ng/ml IL-13 for 72 h. (**b**–**e**) Western blot analysis of Beclin-1, LC3 and P62 and densitometric quantification of bands. Values represent the mean±S.E.M. (*n*=3), ***P<0.001 *versus* normal control. (**f** and **g**) Real-time PCR analysis of miR-34 and miR-449 expression. Values represent the mean±S.E.M. (*n*=3), *P<0.05, **P<0.01, ***P<0.001 *versus* control. (**h**–**j**) Western blot analysis of Nur77 and Bcl-2 and densitometric quantification of bands. Values represent the mean±S.E.M. (*n*=3), ***P<0.001 *versus* control. (**k**) Co-immunoprecipitation analysis of the interaction between Beclin-1, Bcl-2 and Nur77

**Figure 3:** miR-34/449 overexpression suppressed IL-13 induced autophagy by modulating Nur77 subcellular localization via IGFBP-3. BEAS-2B cells were transfected with miR-34/449 mimics or scrambled control mimics and (**a** and **b**) Real-time PCR show the expression of miR-34 (**a**) and miR-449 (**b**) after transfected with miR-34 and miR-449 mimics for 72 h. Values are represented as mean±S.E.M. (*n*=5), ***P<0.001 *versus* control. (**c**–**k**) BEAS-2B cells overexpressing miR-34/449 were treated with or without IL-13 for 72 h (**c**,**d**) Western blot analysis of IGFBP-3 expression and densitometric quantification. Values represent the mean±S.E.M. (*n*=3), *P<0.05, ***P<0.001 *versus* control. ^###^*P*<0.001 *versus* IL-13 group. (**e**–**g**) Western blot analysis of phospho-Akt and total Akt and densitometric quantification of bands. Values represent the mean±S.E.M. (*n*=3), *P<0.05, ***P<0.001 *versus* Control. ^#^*P*<0.05, ^###^*P*<0.001 *versus* IL-13 group. (**h**–**j**) Subcellular distribution of Nur77 analyzed by western blotting. GAPDH was used as the loading control for the total fraction, whereas PARP was used as the loading control for the nuclear fraction. Bar graphs show the quantification of bands by densitometry. Values represent the mean±S.E.M. (*n*=3), *P<0.05, **P<0.01, ***P<0.001 *versus* control. ^#^*P*<0.05, ^###^*P*<0.001 *versus* IL-13 group. (**k**) Representative immunofluorescence images showing the subcellular distribution of Nur77 [Nur77: green; nucleus: DAPI (blue)]

**Figure 4:** miR-34/449 overexpression attenuated autophagy-related fibrosis. BEAS-2B cells transfected with or without miR-34 and miR-449 mimics were treated with or without 3-MA (200 *μ*M) for 1 h before induction with IL-13 for 72 h. (**a**–**d**) Western blot analysis of Beclin-1, LC3 and P62 and densitometric quantification of bands. Values represent the mean±S.E.M. (*n*=3), *P<0.05, **P<0.01, ***P<0.001 *versus* control. ^##^*P*<0.01, ^###^*P*<0.001 *versus* IL-13 group. (**e**–**i**) Western blot analysis of collagen I, collagen III, bFGF and *α*-SMA, and densitometric quantification of bands. Values represent the mean±S.E.M. (*n*=3), *P<0.05, **P<0.01, ***P<0.001 *versus* control. ^##^*P*<0.01, ^###^*P*<0.001 *versus* IL-13 group

**Figure 5:** miR-34/449 overexpression attenuated autophagy-related inflammation. BEAS-2B cells transfected with or without miR-34 and miR-449 mimics were treated with or without 3-MA (200 *μ*M) for 1 h before induction with IL-13 for 72 h. (**a**–**d**) Western blot analysis of the inflammatory factors TNF-*α*, IL-5 and IL-6 and densitometric quantification of bands. Values represent the mean±S.E.M. (*n*=3), *P<0.05, **P<0.01, **P<0.01, ***P<0.001 *versus* control. ^###^*P*<0.001 *versus* IL-13 group. (**e** and **f**) Western blot analysis of NF*κ*B and densitometric quantification. Values represent the mean±S.E.M. (*n*=3), *P<0.05, ***P<0.001 *versus* control. ^#^*P*<0.05, ^###^*P*<0.001 *versus* IL-13 group

**Figure 6:** IGFBP-3 is a target of miR-34/449. (**a**) Sequence alignment between miR-34/449 and the 3′-UTR of human IGFBP-3. Complementary bases between the sequences are shown in red. The sequence of the mutant MALAT1 construct is also shown. (**b**) Dual-luciferase reporter assay of BEAS-2B cells co-transfected with IGFBP-3 3′-UTR-WT or IGFBP-3 3′-UTR-Mut, and miR-34 mimic or miR-NC. Data are presented as the mean±S.D. from six separate experiments. ***P<0.01. (**c**) Dual-luciferase reporter assay of BEAS-2B cells co-transfected with IGFBP-3 3′-UTR-WT or IGFBP-3 3′-UTR-Mut and miR-449 mimic or miR-NC. Data are presented as the mean±S.D. from six separate experiments. ***P<0.01

**Figure 7:** miR-34/449 overexpression suppressed OVA-induced airway remodeling by decreasing autophagy-induced airway inflammation and fibrosis *in vivo*. Airway inflammation was induced in mice by sensitization and treatment with OVA. (**a**–**c**) enzyme-linked immunosorbent assay (ELISA) analysis of the expression of the inflammatory factors TNF-*α*, IL-5 and IL-6 in BALF. Values represent the mean±S.E.M. (*n*=3), ***P<0.001 *versus* control. ^###^*P*<0.001 *versus* OVA group. (**d**) Analysis of pulmonary fibrosis by Masson’s trichrome staining of lung tissues, (original magnification, × 200). (**e**) Immunohistochemical analysis of *α*-SMA expression in lung tissues (magnification, × 200). (**f**) Immunofluorescence analysis of TGF-*β* expression in lung tissues. Nuclei were stained with DAPI (blue) (magnification, × 100). (**g**–**k**) Western blot analysis of bFGF, collagen I, collagen III and *α*-SMA, and densitometric quantification. Values represent the mean±S.E.M. (*n*=3), *P<0.05, **P<0.01, ***P<0.001 *versus* control. ^##^*P*<0.01, ^###^*P*<0.001 *versus* OVA group

**Figure 8:** miR-34/449 overexpression promoted Nur77 nuclear translocation and suppressed autophagy by downregulating IGFBP-3 *in vivo*. Airway inflammation was induced in mice by sensitization and treatment with OVA. (**a**) Representative immunofluorescence images showing the subcellular distribution of Nur77 (magnification, × 400). (**b**–**e**) Western analysis of IGFBP-3, Nur77 and NF*κ*B, and densitometric quantification of bands. Values represent the mean±S.E.M. (*n*=3), *P<0.05, ***P<0.001 *versus* control. ^###^*P*<0.001 *versus* OVA group. (**f**–**i**) Western blot analysis of Beclin-1, LC3 and P62, and densitometric quantification of bands. Values represent the mean±S.E.M. (*n*=3), *P<0.05, **P<0.01, ***P<0.001 *versus* control. ^#^*P*<0.05, ^##^*P*<0.01, ^###^*P*<0.001 *versus* OVA group

**Table 1:** Demographic characteristics and serum cytokine levels

**Characteristics/cytokines**	**Healthy control subjects**	**Asthmatic patients**
*No. of patients*		
	10	46
		
*Sex*		
Male	4	18
Female	6	28
		
*Age (year)*		
	50±12.82	50±14.92
*Height (cm)*		
	165.13±7.32	163.24±8.13
		
*Weight (Kg)*		
	67.35±19.24	65.29±13.29
		
*Smoking*		
Current	2	6
Never smoked	5	34
Ex-smoker	3	6
		
*Age at onset of asthma (year)*		
	0	37.33±17.59
		
*Duration of asthma (year)*		
	0	12.2±13.98
		
*Asthma severity*		
Mild	0	13
Moderate	0	12
Severe	0	21
		
*IgE sensitization (IU/ml)*		
	72±32.52	168.29±141.72***
		
*B-Eos (× 10*^*9*^*/l)*		
	0.12±0.43	0.43±0.37***
		
*Inflammatory factor (pg/ml)*		
IL-5	111.56±16.62	251.13±52.38***
IL-6	149.60±29.29	306.50±33.43***
IL-13	32.06±11.43	64.95±16.76***
TNF-*α*	27.00±8.27	49.86±10.27***
		
*Fibrosis related protein (pg/ml)*		
bFGF	236.88±49.44	665.88±175.23***
IGFBP-3	122.96±88.00	632.92±222.35***
TGF-*β*	250.18±48.79	670.93±143.57***

Abbreviations: B-Eos, blood eosinophils; bFGF, basic fibroblast growth factor; IgE, immunoglobulin E; IGFBP-3, insulin-like growth factor (IGF) binding proteins 3; IL, interleukin; TGF-*β*, transforming growth factor. ***P<0.001 against the healthy control values. Data are expressed as mean±S.D.
